# The Incidence of Septic Pulmonary Embolism in Patients with *Klebsiella pneumoniae* Liver Abscess: A Systematic Review and Meta-analysis

**DOI:** 10.1155/2022/3777122

**Published:** 2022-04-15

**Authors:** Yunan Wang, Hairui Wang, Zhaoyu Liu, Zhihui Chang

**Affiliations:** Department of Radiology, Shengjing Hospital of China Medical University, Shenyang, China

## Abstract

*Background*: Septic pulmonary embolism (SPE) is an associated complication of *Klebsiella pneumoniae* liver abscess (KPLA). However, previous studies have reported that its incidence varies widely. We conducted a systematic review and meta-analysis to investigate the incidence of SPE in patients with KPLA. We further analyzed their clinical and computed tomography (CT) features. *Methods*: Two researchers reviewed PubMed, EMBASE, Web of Science, and Cochrane Library databases to identify the articles that reported SPE in patients with KPLA. The search was conducted from the date of establishment of each database up to January 2021. After screening the articles and extracting the data, we used Review Manager 5.3 for analysis and processing. *Results*: We selected six articles that included 1,158 patients with KPLA. Of these, 70 patients had SPE. The pooled incidence of SPE was 6% (95% confidence interval, 3%–9%). Among patients with SPE, 85% were men, 72% had diabetes, and 52% displayed the feeding vessel sign on the chest CT. The mortality rate was 12%. Quality assessment revealed that half of the included studies had a high quality. *Conclusion*: The pooled incidence of SPE in patients with KPLA was 6%. Men and patients with diabetes were more prone to SPE. For patients with KPLA who had SPE as an associated complication, the mortality rate was approximately 12%.

## 1. Introduction

Liver abscess is a common infectious disease caused by bacteria, fungi or parasites. *Escherichia coli* had always been the most common causative agent implicated in liver abscess. However, since the mid-1980s, an increasing number of cases of *Klebsiella pneumoniae* liver abscess (KPLA) have been reported, especially in Asia [1–4]. Patients with KPLA are prone to migratory infections, such as septic pulmonary embolism (SPE), endogenous endophthalmitis, and meningitis, a condition known as invasive *Klebsiella pneumoniae* liver abscess syndrome (IKPLAS) [5].

Septic pulmonary embolism (SPE) is a non-thrombotic, pathogen-containing thrombus causing bacterial embolism in the pulmonary vessels derived from a primary infection site via the venous circulation [6]. The reported incidence of SPE in patients with KPLA varies from 2.7% to 16.3% [6–11]. However, its prevalence remains unclear due to the paucity of large sample or population-based studies. Meanwhile, awareness about SPE among clinical staff is inadequate. In clinical practice, radiologists rarely diagnose SPE, and some may mistake it for malignant lung metastases. Respiratory physicians are often unable to distinguish SPE from community-acquired pneumonia. Therefore, the diagnosis and treatment of SPE is often delayed [12, 13].

However, SPE induced by KPLA can rapidly progress from light respiratory symptoms to respiratory failure and septic shock. Further, it carries a higher mortality rate than KPLA alone [6–8]. A thorough understanding of the clinical and radiological characteristics of SPE will aid its diagnosis and treatment. Therefore, this study was aimed at evaluating the incidence of SPE in KPLA patients by reviewing previous related studies. Further, we discuss the clinical and computed tomography (CT) features of SPE associated with KPLA.

## 2. Method

We conducted the systematic review in accordance with the guidelines of the Cochrane Handbook for Systematic Reviews of Intervention [14] and the Preferred Reporting Items for Systematic Reviews and Meta-Analysis (PRISMA) guidelines [15].

### 2.1. Literature Search

Two researchers reviewed the PubMed, EMBASE, Web of Science, and Cochrane Library databases to identify articles regarding SPE in patients with KPLA. We included articles from the time each database was established up to January 2021, using combinations of the following keywords: “septic pulmonary embolism,” “septic pulmonary emboli,” “liver abscess,” “hepatic abscess,” “Klebsiella,” and “pyogenic liver abscess.”

Two authors independently reviewed the articles based on the inclusion and exclusion criteria listed below. Any differences in opinions regarding selection of the articles were resolved by discussion with a third author, who made the final decision. Finally, the references of the selected studies were screened to identify any other potentially relevant studies for inclusion.

### 2.2. Selection of Studies

The inclusion criteria for the studies were as follows: (1) Patients with liver lesions on CT, (2) patients for whom pus was extracted during drainage or diagnostic aspiration and the pus or blood culture indicated the presence of *Klebsiella pneumoniae*, (3) studies that included fifty or more patients with KPLA, and (4) the studies for which the number of cases of SPE in patients with KPLA was stated. We used the following exclusion criteria: (1) Studies wherein SPE was only investigated in a particular subgroup of patients with KPLA, or (2) studies wherein the concept of SPE was not clearly described.

### 2.3. Characteristics of Included Studies

We included six studies [6–11] (Figure 1), which comprised of 1,158 patients with KPLA, 70 of whom developed SPE. The studies were conducted in four different geographic locations: China, Taiwan [6, 7, 10]; China, mainland [8]; Singapore [9]; and South Korea [11]. All the studies were published from 2008 to 2015. The number of patients with KPLA in each study ranged from 92 [9] to 355 [7]. All studies were retrospective in their methodology (Table 1).

### 2.4. Extraction of Data

Two authors independently extracted and entered the data from each included study in standardized Microsoft Excel sheets. The same authors examined the data, and consensus was reached for any discrepancy by reviewing the study. The following information was extracted from each article: characteristics of the study (year, authors, place, type of study, and time period) and assessment of SPE (number of SPE cases and clinical and radiological features).

### 2.5. Assessment of the Quality of the Included Studies

Two authors independently assessed each included study for the methodological quality. A predefined scale that included the following eight items was used for assessment, with “yes” and “no” as options for the answers: (1) KPLA represented the entire population and not a sample thereof, (2) unbiased sampling frame, (3) adequate sampling, (4) the criteria for diagnosing KPLA were described, (5) SPE was detected using standard protocols, (6) SPE was assessed by unbiased personnel, (7) the criteria for diagnosing SPE were described, and (8) outcomes were reported for 70% or more of the patients with KPLA. Each positive answer was assigned one point. We defined the following ranges to qualitatively classify the overall quality of the research: 0–4 = poor quality; 5–6 = fair quality; and 7–8 = high quality [16].

### 2.6. Statistical Analysis

Considering the expected heterogeneity in effect sizes [17], a pooled estimate of the incidence of SPE in patients with KPLA was performed using a random-effects model based on the method described by Der Simonian and Laird [18]. We assessed the heterogeneity among the included studies using forest plots, which graphically represented the effect size with the 95% confidence interval (CI). Further, a two-tailed (*p* < 0.05) was considered statistically significant [19]. We used the Cochran Q test to assess the statistical heterogeneity and quantified it using the *I*^2^ index.

## 3. Results

### 3.1. Incidence of SPE in KPLA

Seventy patients had SPE in the six selected studies. The lowest incidence was 2.7% (9 of 335 patients) and the highest was 7.9% (15 of 92 patients). Using the random-effects model, the pooled incidence rate of SPE in patients with KPLA was 6% (95% CI, 3%–9%) (Figure 2). The studies had high (*I*^2^ = 76%) and significant (*p* < 0.001) heterogeneity of incidence.

### 3.2. Clinical and Radiological Features of SPE

Three studies included data on the sex of patients and the occurrence of SPE. A consolidation analysis revealed that male patients constituted 85% of the patients who developed SPE (95% CI, 69%–101%) (Figure 3(a)).

Patients with diabetes are at high risk for KPLA. We conducted a consolidated analysis to analyze the association between diabetes and SPE, which revealed that 72% of patients with SPE had diabetes (95% CI, 51%–93%). This indicates a close association between diabetes and SPE (Figure 3(b)).

Mortality is a crucial prognostic indicator, and our analysis revealed a mortality rate of 12% in patients with KPLA complicated by SPE (95% CI, 1%–25%) (Figure 3(c)).

Previous studies have indicated that the feeding vessel sign (FVS) is a typical radiological finding in SPE. In this meta-analysis, 52% of patients with SPE displayed FVS (95% CI, 22%–82%) (Figure 3(d)).

### 3.3. Assessment of the Quality of each Study

Three studies were assigned as high quality [6–8], three as fair quality [9–11], and no studies as poor quality (Table 2).

## 4. Discussion

To the best of our knowledge, this is the first systematic review and meta-analysis that evaluated the incidence of SPE in patients with KPLA. For the six studies included in our study, the incidence of SPE in 1,158 patients with KPLA was 6% (95% CI, 3%–9%). Although few studies reported multiple neutrophils and foam tissue cells as the pathologic findings of SPE [20], percutaneous needle aspiration biopsy is difficult in clinical practice. The diagnosis of SPE is primarily based on assessment of the clinical and radiological features. It is difficult to distinguish SPE from other pulmonary diseases. Therefore, we summarized the clinical and radiological manifestations of SPE to determine and treat it in a timely and accurate manner.

Our analysis revealed that 85% of KPLA patients with SPE was men and 72% had diabetes. Several studies on bacterial pathogenesis have documented that the capsular polysaccharide serotypes K1 and K2 of *Klebsiella pneumoniae* are the key microorganism virulence factors that contribute to the development of septic metastatic infection [21, 22]. Lin et al. further identified that neutrophil-mediated phagocytosis of *Klebsiella pneumoniae* is impaired in diabetic patients with poor glycemic control, which contributes to the development of metastatic infection in liver abscesses [23]. Therefore, diabetes is an important risk factor for cases of KPLA that are complicated by SPE. The two most common symptoms of SPE are fever and shortness of breath, which are not particularly different from those of other respiratory infections. Therefore, clinicians should be alert about the possibility of SPE when KPLA patients with diabetes or those who are male present with respiratory symptoms.

SPE is suspected in other lung infections or tumors; hence, it is necessary to clarify the CT features of SPE. The most common CT features of SPE include FVS, multiple nodules, peripheral wedge-shaped shadows, halo sign, and pleural effusion [6, 8, 11]. These features are complex and may coexist. In this study, we found FVS in approximately 52% of the KPLA patients with SPE. In a previous study with 168 cases of KPLA patients with SPE, the cause of SPE included drug addiction, infective endocarditis, intravascular indwelling catheters, and liver abscess. Herein, 37 patients (27.6%) displayed FVS signs on the CT [24]. However, in the current study, we observed 52% incidence of FVS, which possibly indicates that the incidence of FVS is higher in patients with KPLA-induced SPE. Although the pulmonary nodules or wedge-shaped lesions caused by septic emboli are due to the embolization of the small branches of the pulmonary arteries, the conventional CT techniques followed presently cannot detect these arteries. Reports have shown that pulmonary veins, and not pulmonary arteries, are involved in FVS. The most likely transfer route of SPE is that *Klebsiella pneumoniae* invades the adjacent hepatic veins, resulting in thrombophlebitis. It then enters the inferior vena cava, subsequently invading the lung parenchyma via the pulmonary artery, and finally forms SPE [8].

The pooled mortality rate of KPLA with SPE was 12% in the current study, and the reported mortality rate of KPLA ranged from 5.4% to 6.1% [7, 10]. Six patients with SPE died in the three included studies. The main causes of death were respiratory failure and septic shock. Three patients had extrapulmonary metastases, of which two had septic metastatic meningitis and one had septic metastatic pericarditis. If SPE is not controlled in time, it might cause respiratory failure and endanger the life of the patient. In addition, KPLA patients with SPE are more likely to develop extrahepatic disseminated infections and septic shock [8], which cause high mortality in SPE patients.

Many studies have reported the incidence of “pulmonary abscess” and “pulmonary infection” in patients with KPLA without using the term “SPE” [25, 26]. This may result in the underestimation of the true incidence of SPE in patients with KPLA. In addition, some nodules are too small to appear on chest X-rays, and they can only be identified on chest CT scans—this constitutes another reason for the underestimation of the incidence of SPE in patients with KPLA. Therefore, we recommend routine chest CT scans instead of chest X-rays for patients with liver abscesses to facilitate earlier identification of SPE.

Our study had several limitations. First, the available literature and the sample size were limited and only three of the six included studies were of high quality. Second, all the studies included had a retrospective design and thus had inherent biases and limitations. In addition, these studies led to considerable heterogeneity in the incidence of SPE in KPLA in different periods and populations.

In summary, this meta-analysis estimated the incidence of SPE in patients with KPLA at 6%. SPE mostly occurred in patients with KPLA who had diabetes or were male. The most relevant CT feature of SPE was FVS. KPLA accompanied by SPE has a poor prognosis. However, considering that only half of the articles included in this study were of high quality, our conclusions should be interpreted with caution. Future studies with larger samples are needed to provide further evidence.

## Figures and Tables

**Figure 1:** A schematic flowchart of the Preferred Reporting Items for Systematic Reviews and Meta-Analyses (PRISMA) guidelines. Six studies were finally selected.

**Figure 2:** The incidence of septic pulmonary embolism (SPE) in patients with *Klebsiella pneumoniae* liver abscess (KPLA). A pooled estimate of the incidence of SPE in patients with KPLA revealed that the overall incidence was 6% (95% CI, 3%–9%). There was considerable and significant heterogeneity (*p* < 0.01, *I*^2^ = 76%).

**Figure 3:** The clinical and imaging features of SPE. (a) 85% patients with SPE were male (95% CI, 69%–101%). There was fair and moderate heterogeneity (*p* = 0.11, *I*^2^ = 54%). (b) 72% patients with SPE had diabetes mellitus (95% CI, 51%–93%). There was considerable and substantial heterogeneity (*p* < 0.10, *I*^2^ = 64%). (c) The pooled mortality rate of *Klebsiella pneumoniae* liver abscess (KPLA) with SPE was 12% (95% CI, –1%–25%). There was considerable and moderate heterogeneity (*p* < 0.10, *I*^2^ = 43%). (d) 52% patients with SPE had the feeding vessel sign (95% CI, 22%–82%). There was considerable and significant heterogeneity (*p* < 0.10, *I*^2^ = 81%).

**Table 1:** Characteristics of included studies.

Study	Place	Period of study	Study design	Setting	KP				SPE			
					No.	Mean years	Males (%)	DM (%)	No.	Mean years	Males (%)	DM (%)
Chou et al. [6]	China, Taiwan	2005.01–2013.12	RC	1 hospital	221	NR	NR	NR	14	59.6	71.4	86
Alsaif et al. [9]	Singapore	2003.07–2010.07	RC	1 hospital	92	56.5	72.8	48.9	15	NR	NR	NR
Yoon et al. [11]	South Korea	2004–2011	RC	1 hospital	161	61.2	60.9	27.3	6	NR	NR	NR
Yang et al. [7]	China, Taiwan	1999.01–2005.12	RC	1 hospital	355	NR	NR	NR	9	56	77.8	66.7
Lee et al. [10]	China, Taiwan	2001–2002	RC	1 hospital	110	61.8	53.6	60.9	5	NR	NR	NR
Chang et al. [8]	China, mainland	2010.01–2015.5	RC	1 hospital	239	NR	NR	NR	21	52.38	95.28	52.38

DM: diabetes mellitus; KP: *Klebsiella pneumoniae* liver abscess; NR: not reported; RC: randomized controlled; SPE: septic pulmonary embolism.

**Table 2:** Assessment of the quality of each study.

Study	KPLA represented the entire population	Unbiased sampling frame	Adequate sampling	The criteria for diagnosing KPLA were described	SPE was detected using standard protocols	SPE was assessed by unbiased personnel	The criteria for diagnosing SPE were described	Outcome reported for 70% or more of patients with KPLA	Score
Chou et al. [6]	Yes	Yes	Yes	No	Yes	Yes	Yes	Yes	7
Alsaif et al. [9]	Yes	Yes	Yes	Yes	No	No	No	Yes	5
Yoon et al. [11]	Yes	Yes	Yes	Yes	No	No	No	Yes	5
Yang et al. [7]	Yes	Yes	Yes	Yes	Yes	Yes	Yes	Yes	8
Lee et al. [10]	Yes	Yes	Yes	Yes	No	No	No	Yes	5
Chang et al. [8]	Yes	Yes	Yes	No	Yes	Yes	Yes	Yes	7

KPLA: *Klebsiella pneumoniae* liver abscess; SPE: septic pulmonary embolism.

## Data Availability

All data generated or analyzed during this study are included in this published article and its supplementary information files.
